# Integrated Network Pharmacology and Gut Microbiota Study on the Mechanism of Huangqin Decoction in Treatment Diabetic Enteritis

**DOI:** 10.1155/2022/5080191

**Published:** 2022-04-07

**Authors:** Xiaomin Xu, Cheng Fang, Fang Lu, Shumin Liu

**Affiliations:** ^1^Heilongjiang University of Chinese Medicine, Harbin 150040, China; ^2^Drug Safety Evaluation Center of Heilongjiang University of Traditional Chinese Medicine, 150040, China; ^3^School of Continuing Education, Heilongjiang University of Traditional Chinese Medicine, China

## Abstract

**Objective:**

Using network pharmacology and gut microbiota sequencing to investigate the probable mechanism of Huangqin decoction in the treatment of Diabetic enteritis (DE).

**Methods:**

The mechanism of Huangqin decoction on DE was studied by combining network pharmacology and gut microbiota sequencing analysis. The core components and possible targets of Huangqin decoction were analyzed by network pharmacology. The effect of Huangqin decoction on microorganisms was investigated by gut microbiota sequencing.

**Results:**

The results of gut microbiota sequencing analysis showed the abundance of TM7, Tenericutes, Chloroflexi, Cyanobacteria, Acidobacteria, WS6, [Prevotella], Helicobacter, Prevotella, Lactococcus, and Anaeroplasma in the Huangqin decoction group had a significant downward. Using a network pharmacology-related database, 141 main active components of Huangqin decoction were identified, as well as 256 corresponding component targets and 1777 corresponding disease targets; the disease targets and component targets were mapped, and topological analysis was used to determine the potential of Huangqin decoction in the treatment of DE. There were 156 targets, of which the top 20 genes were selected for GO and KEGG. The KEGG results showed that 134 pathways were enriched, which was partially consistent with the metabolic pathways of gut microbiota sequencing analysis.

**Conclusion:**

The results show that Huangqin decoction can inhibit the expression of inflammatory factors and related inflammatory pathways in intestinal epithelial cells, thereby regulating the structure of intestinal flora. Using picurst2 for functional prediction and metabolic pathway statistics, seven metabolic pathways were obtained consistent with gut microbiota sequencing, and the NOD-like receptor signaling pathway may be its potential molecular mechanism. These results help to understand the mechanism of Huangqin decoction on DE and provide the theoretical basis for further study of Huangqin decoction.

## 1. Introduction

Diabetes mellitus is a widespread disease. According to the International Diabetes Federation, it affects 463 million people worldwide with an increasing prevalence [1]. Diabetes is an important public health burden, mainly because of its cardiovascular, renal, and neurological complications. Furthermore, many people with diabetes have upper gastrointestinal (GI) symptoms as well as motor abnormalities. Up to 50% of individuals with type 1 and type 2 diabetes suffer dyspepsia and gastroparesis or are asymptomatic in certain cases, impacting 50% of delayed gastric emptying [2]. These two clinical symptoms share similar pathogenic mechanisms, including autonomic neuropathy, changes in the enteric nervous system, and histological abnormalities. Dyspeptic symptoms are common in people with diabetes, and they are part of the so-called diabetic bowel disease [3]. Studies have shown that the intestinal environment of T2DM patients is in a chronic low-grade inflammatory response [4]. Some literature has shown that intestinal flora is closely related to the systemic chronic inflammatory response. Oral antibiotics can regulate the intestinal flora of diabetic patients, reduce inflammation in the body, and improve the phenotype of T2DM. It is worth noting that oral antibiotics can inhibit intestinal flora. Antibiotics may also cause damage to the beneficial intestinal flora, leading to an imbalance of intestinal flora, which may have adverse effects on diabetic patients [5].

Huangqin decoction is a traditional Chinese medicine formula in the classic Chinese medical book “Treatise on Febrile Diseases” written by Zhang Zhongjing of the Eastern Han Dynasty. It has a history of nearly 1800 years and is widely used in the clinical treatment of intestinal diseases such as ulcerative colitis [6–9]; it is made by frying four traditional Chinese medicines: Scutellaria baicalensis, Paeonia lactiflora, jujube, and licorice. In Huangqin decoction, according to traditional Chinese theory, Scutellariae is the king, which is bitter, cold, hardy yin, and clears heat in the interior; Shaoyao is the minister in this medicine, slightly bitter and sour, relieving acute pain, astringing yin, and nourishing. Preserving yin to stop dysentery is essential for treating dysentery; licorice and jujube benefit qi and neutralize the middle. Adjust and supplement the righteousness [10]. Scutellaria baicalensis decoction is precise and has less medicinal flavor. Scutellaria baicalensis has the effect of clearing heat and relieving dysentery, Paeonia lactiflora has the functions of astringing Yin, nourishing and relieving pain, and licorice and jujube can help neutralize the stomach, invigorate the spleen and stop diarrhea, and nourish qi and nourish liquid. On one side, it also has the methods of clearing heat, detoxifying, drying dampness, cooling blood, and nourishing sweetness. Therefore, it is called “the ancestral prescription for treating dysentery.”

Pharmacological studies have shown that Huangqin decoction has anti-inflammatory, antibacterial, analgesic, antipyretic, sedative, and other effects. In recent years, with extensive research on Huangqin decoction, it has been used to treat acute lung injury, colon cancer, gastric cancer, leukemia, and other diseases according to its anti-inflammatory, antiproliferation, and mucosal protective effects [11–14]. It is mainly used to treat intestinal inflammation and is considered to have a significant effect on intestinal inflammation and mucosal protection in the intestinal tract. It was found that gut flora played a critical role in the investigation of its mechanism of action [15]. It was discovered that the intestinal flora can not only act directly on the intestinal mucosa, exerting anti-inflammatory and mucosal protective effects, but can also affect the metabolism of the components in Huangqin decoction, metabolizing the more difficult-to-absorb components such as baicalin into the more easily-absorbable components such as baicalein, thereby augmenting the therapeutic effect of Huangqin decoction [7]. Simultaneously, as experimental animal research has progressed and clinical use of Huangqin decoction has expanded, it has been discovered that it has a favorable therapeutic impact in the treatment of ulcerative colitis and other disorders [16].

Therefore, based on network pharmacology and gut microbiota, this study will investigate the mechanism of Huangqin decoction in the treatment of DE.

## 2. Materials and Methods

### 2.1. Experimental Materials

Experimental materials are as follows: Scutellaria baicalensis; Baishao; Jujube; Licorice (all purchased from Hebei Quantai Pharmaceutical Co., Ltd.); DNeasy PowerSoil Kit (QIAGEN, Netherlands); Quant-iT PicoGreen dsDNA Assay Kit (Invitrogen, USA); Agcout AMPure Beads (Beckman Coulter, USA); PicoGreen dsDNA Kit (Invitrogen, USA); CD45 antibody (Santa, USA); PV9004 secondary antibody (Zhongshan, Beijing); DAB chromogen (Zhongshan, Beijing); Quantifluor-ST fluorometer (Promega); high-throughput sequencer (Illumina, USA); low-temperature medical freezer (Haier Co., Ltd.); gdsAUTO520 gel imaging system (BG Corp., USA); DYY-6C electrophoresis instrument (ABI, USA); paraffin embedding machine (LeicaEG1150H); paraffin microtome (Leica RM 2125 RTS); paraffin microtome (Leica HI1220); and fluorescence microscope (OLYMPUS DP80).

Preparation of Huangqin decoction: weigh the decoction pieces of Radix Scutellariae, Radix Paeoniae Alba, jujube, and licorice in the ratio of 3 : 2 : 2 : 2, add 10 times the total weight of water, soak for 30 minutes, decoct for 1 hour, filter the filtrate, add 8 times the volume of water to decoct for 1 hour, filter the filtrate, combine the two filtrates, and concentrate to 1.5 g/mL, and the low-dose concentration of Huangqin decoction is 0.5 g/mL.

### 2.2. Experimental Animals

The 48 male db/db mice and 8 db/m mice were purchased from Aiermaite Technology Co., Ltd. (animal certificate number: no. 202009670). The mice were housed in a single cage in a clean-grade barrier system with free food. Drinking water, temperature controlled at 20-26°C, humidity controlled at 40-70% kept 12/12 hours of animal lighting alternating in the light and dark cycle, changing cages, and bedding once a week. All animal experiment-related operations were followed relevant regulations of the Laboratory Animal Ethics Committee of Heilongjiang University of Traditional Chinese Medicine. The db transgenic mice were adaptively fed for one week after purchase, and 2 random blood glucose tests were performed. db/db mice with blood glucose values higher than 11.1 mol/L were selected for grouping and divided into a model group and a low-dose Huangqin decoction group (3.75 g/kg) and Huangqin decoction high-dose group (11.25 g/kg), and db/m mice were the blank group; after grouping, the mice were administered once a day, and the administration volume was 7.5 mg/kg for 8 weeks.

### 2.3. Sample Collection and Processing

Before the sacrifice, body weights of each mice in tested groups were recorded. After the mice were sacrificed, the cecum contents were taken and placed in a sterile tube in time. After sealing, they were quickly frozen with liquid nitrogen and transferred to a refrigerator at -80°C for storage for subsequent analysis. The epididymal adipose tissue was stored at −75°C. A small portion of the liver tissue was placed in formaldehyde solution of 4% concentration, and the remaining liver tissue was stored at −80°C for further tests. Similarly, intestinal tissues were collected and frozen for further experimental purposes.

### 2.4. H&E Staining

The cecal tissues of mice were dehydrated and waxed; slice and paste the cut film on the cover glass to dry; before staining, the paraffin in the section must be removed with xylene, then through high concentration to low concentration alcohol, and finally, into distilled water to dye; put the slices that have been put into distilled water into hematoxylin aqueous solution for dyeing for several minutes; color separation in acid water and ammonia water for several seconds, respectively; after washing with running water for 1 h, add distilled water for a moment; dehydrate in 70% and 90% alcohol for 10 minutes, respectively; add alcohol eosin staining solution for 2~3 minutes.

### 2.5. Immunohistochemistry

According to the consensus criteria developed for type 1 diabetes, an individual can be diagnosed with insulitis when ≥15 CD45^+^ cells are found within the parenchyma or in the islet-exocrine interface in ≥3 islets. The changes of expression of CD45 in the cecal tissue of diabetic cardiomyopathy mice were taken from the cecum tissues, fixed with wax blocks, and then, cut and sealed for 78 degrees in the oven. After the morning was taken out, the xylene was fixed for 10 min, dehydrated with alcohol, then dehydrated 5~10 min; distilled water was washed for 2 times, 3~5 min/times, 3% H_2_O_2_ blocked 10 min; distilled water was cleaned 2 times, 3~5 min/times. Citric acid repair (add the tissue after boiling water, stop heating after steam, open the air valve after 2~3 minutes, open the cover after 7 minutes, and take out the tissue), cool for about 50 minutes, wash the tissue with PBS for 3 times after cooling, 5 min/time, and add primary antibody (100 *μ* 50). Incubate overnight at 4°C, wash PBS for 3 times the next day, 5 min/time, and add secondary antibody (100 *μ* 50). Incubate at room temperature for 30 min, wash with PBS for 3 times, 5 min/time, DAB color development for 5-10 minutes (block the color development after observing the color development under the microscope), hematoxylin reappears for 1 min after washing with water for 3-5 minutes, wash with water for 10-15 minutes after observing the dyeing degree under the microscope (if it is not ideal, it can be dyed repeatedly), dehydrate and dealcoholic for 2-3 min/time after washing with distilled water, and finally, seal the neutral gum in the incubator at 87°C for 2-3 days. The film is taken under the microscope and stored in the computer.

### 2.6. 16S rRNA Gene Sequencing

#### 2.6.1. DNA Extraction from Stool Samples

The Dneasy powerOil kit of QIAGEN company was used for extraction and DNA detection. The absorbance values of the extracted DNA were measured at 260 nm and 280 nm, respectively, by fluorescence spectrophotometer, the concentration of DNA was calculated, and the quality of DNA was detected by agarose gel electrophoresis of 1%. Adjust the concentration of DNA solution according to the results, and then, store the adjusted DNA working solution in a 4°C refrigerator and the storage solution in a -20°C refrigerator.

#### 2.6.2. 16S rRNA Gene Amplicon Sequencing

The v3-v4 region of the 16S rRNA gene of flora was amplified by PCR with forward primer (ACTCCTACGGGAGGCAGCA) and reverse primer (GGACTACHVGGGTWTCTAAT). The sample-specific 7 bp barcode was integrated into primers for multiple sequencing. The PCR component contains 5 *μ*L Q5 reaction buffer (5) ×, 5 *μ*L Q5 high fidelity GC buffer (5) ×, zero point two five *μ*L Q5 high fidelity DNA polymerase (5*μ*)/*μ*L), 2 *μ*L (2.5 mM) dNTPs, 1 *μ*L (10 *μ*M), DNA template solution 2 *μ*L, and ddH2O 8.75 *μ*L. The thermal cycle includes initial denaturation at 98°C for 2 min, then denaturation at 98°C for 15 s, annealing at 55°C for 30 s, extension at 72°C for 30 s, 25 cycles, and final extension at 72°C for 5 min. PCR amplicons were purified with Agcout AMPure Beads and quantified using PicoGreen dsDNA detection kit (Invitrogen, Carlsbad, CA, USA). After a single quantification step, equal amounts of amplified products were collected, and paired-end 2 × 300 bp sequencing was performed using the Illumina MiSeq platform and MiSeq Kit v3 at Shanghai Parsono Biotechnology (Shanghai, China) Co., Ltd.

#### 2.6.3. Sequencing Data Processing

The data obtained were dedried by DADA2 and Vsearch using the Parsono gene cloud platform. The R language script was used to calculate the high-quality sequences' length distribution in all samples. The QIIME2 analysis software was used to perform species taxonomic annotation, taxonomic composition analysis, and diversity analysis, and random forest analysis between multiple groups of samples was used to find the different flora between groups. Finally, the PICRUSt2 analysis software was used to predict functional potential [17].

### 2.7. Data Processing

Statistical analysis was performed using the SPSS 20.0 software. Wilcoxon rank sum test was used to compare the two groups of samples, and Kruskal Wallis test was used to compare the three groups of samples.

### 2.8. Network Pharmacology Analysis

Using the TCMSP database, the active components of Huangqin decoction were screened under the conditions of oral absorption and utilization (OB) ≥30% and drug class (DL) ≥ 18%, and the screened components were supplemented in combination with literature reports. The obtained components were sequentially imported into the TCMSP database, the target was predicted, and the protein name of the relevant target was obtained, which was imported into the Uniprot database, and the gene name was transformed to obtain the relevant target of traditional Chinese medicine. The GeneCards database was used to search “DE,” and the intersection of the disease target and the drug target was used as the prediction target of the drug acting on the disease. Gene and protein names were standardized using the Uniprot database (http://www.uniprot.org/). The target information of the interaction between Huangqin decoction and DE obtained above was imported into the STRING database (https://string-db.org/) to obtain the relationship between potential targets. The Cytoscape v3.8.2 software was used to visualize and analyze the protein interaction analysis results of the STRING database to construct a protein-protein interaction network. The clusterProfiler package in R language was used to perform GO functional annotation enrichment analysis and KEGG pathway analysis for common targets. The enriched pathways are the potential pathways for the drug to play a therapeutic role, and a histogram is drawn to visualize it.

## 3. Results

### 3.1. H&E Staining

The degree of damage to the integrity of the intestinal barrier reflects the barrier function of the intestinal mucosa to a certain extent. In this study, the length of the intestinal mucosal villi and the thickness of the muscularis layer were observed by H&E staining to determine the change of the intestinal mucosal barrier function, as shown in Figure 1. H&E staining showed that the villus length and muscle thickness of the intestinal mucosa in the blank group were normal (Figure 1(a)); the villi were shortened, and the muscle layer thickness was decreased in the model group (Figure 1(b)); the symptoms of the Huangqin decoction group were more severe than those of the model group. The villus length was similar to that of the blank group, but the thickness of the muscle layer was still significantly lower than that of the blank group (Figure 1(c)).

### 3.2. Immunohistochemistry

The intestinal mucosa was sectioned, and the differences in leukocyte infiltration were observed by CD45 staining, as shown in Figure 2. In the blank group, only a few CD45+ cells were infiltrated. Compared with the blank group, the infiltration of CD45+ cells in the model group were significantly increased, while that in the Huangqin decoction group was significantly less than that in the model group (Figures 2(a)–2(c)).

### 3.3. 16S rRNA Gene Sequencing

#### 3.3.1. Classification and Analysis of OTUs (Operational Taxonomic Units) of Gut Microbiota in Samples from Each Group

The blank group has a total of 5450 OTUs and 3297 unique OTUs, the model group has a total of 5678 OTUs and 3561 unique OTUs, the Scutellaria baicalensis soup has a total of 5580 OTUs and 3747 unique OTUs, and the three groups have a total of 837 OTUs, as shown in Figure 3. Compared with the blank group, the number of OTUs in the model group was significantly increased; compared with the model group, the number of OTUs in the administration group was significantly downregulated.

#### 3.3.2. Alpha Diversity Analysis of Gut Microbiota in Each Group

As shown in Figures 3(b)–3(d), the diversity of samples in each group is almost saturated, indicating that the sequencing depth is sufficient and the sample size of each group is sufficient to reflect the richness of the community. The biodiversity indexes of the three groups of samples were compared, as shown in Table 1. Compared with the blank group, the intestinal flora Chao1, Faith_pd, Goods_coverage, Observed_species, Pielou_e, Shannon, and Simpson indexes of mice in the model group all showed a downward trend. After the administration of Huangqin decoction, all diversity indices showed a downward trend, as shown in Table 1.

#### 3.3.3. Taxonomic Composition Analysis of Gut Microbiota in Each Group

Through the analysis of Figures 4(a) and 4(b), it is found that Bacteroides and Firmicutes are the most important phyla at the phylum level, followed by tenerictes, Proteobacteria, and actinobacteria. These five phyla account for a very high proportion of the whole phyla and belong to the dominant phyla. Compared with the blank group, in the model group, bacteroidea (54.25% → 43.77%), Firmicutes (38.06% → 47.37%), Firmicutes (2.48% → 5.55%), proteus (2.98% → 0.01%), actinomycetes (0.89% → 0.73%), and Firmicutes/Bacteroidetes ratio in the blank group was 0.70, and Firmicutes/Bacteroidetes ratio in the model group was 1.08. It is suggested that the dominant flora of model group mice and blank group mice has changed significantly in the structure; compared with the model group, the ratio of Firmicutes/Bacteroidetes in Huangqin decoction group was 1.14, suggesting that Huangqin decoction could regulate the dominant flora of db/db mice.

From the subordinate level, through cluster analysis of the absolute dominant bacterial genera in the top 20, find and analyze the relative abundance of different bacterial genera, namely, Bacteroides, oscillospira, anaeroplasma, Lactobacillus, odoribacter Ruminococcus, Desulfovibrio, Lactococcus, dehalobacterium, rikenella, alistipes, adlercreutzia, candidatus_arthromitus, coprococcus Helicobacter, parabacteroides, and Staphylococcus.

#### 3.3.4. Influence of Gut Microbiota on Beta Diversity Analysis

In this study, PCoA analysis was used to investigate the differences in the beta diversity of rat gut microbiota. There was no significant difference in the diversity of bacterial community structure in the blank, model, and Huangqin decoction groups, and the communities in each group fell within their respective ranges, with strong similarity. The results showed that compared with the blank group, the microflora of the mice in the model group were significantly separated, indicating that the beta diversity of the two groups was significantly different. After administration of Huangqin decoction, it tended to the blank group, indicating that the beta diversity of the Huangqin decoction group was similar to that of the normal group. After administration of Huangqin decoction, it had a certain effect on the body of DE mice, as shown in Figure 4(c).

Differences between groups were analyzed by (permutational multivariate analysis of variance (PERMANOVA)). The results showed that the differences in the bacterial community structure diversity within the blank group, the model group, and the Huangqin decoction administration group were significantly smaller than the differences between the groups, suggesting that the blank group, the model group, and the Huangqin decoction administration group had significant effects on the bacterial community structure diversity. There were significant between-group differences, see Table 2.

#### 3.3.5. Gut Microbiota Difference Analysis

Using the method of random forest analysis, we screened the different gut microbiota among the experimental groups. We found that the gut microbiota with differences at the phylum level included deferribacteris, Proteobacteria, tenericutes, Firmicutes, acidobacteria, cyanobacteria, Actinobacteria, Bacteroidetes, fusobacteria, tm7-3, Chloroflexi, and WS6. The gut microbiota with differences at the class level include Mollicutes, epsilon Proteobacteria, deferribacterias, deltaproteobacteria, Actinobacteria, tm7-3, gamma Proteobacteria, bacteroidia, coriobacteria, clostridia, erysipelotrichi, betaproteobacteria, Alphaproteobacteria, synechococcophycedeae, bacilli, [chloracidobacteria], Flavobacteria Chloroflexi,TM7-1, and Fusobacteriia. The gut microbiota with differences at the order level include deferribacteriales, desulfovibrionales, bacillales, actinomyceteales, campylobacterales, bifidobacteria, caulobacterales, enterobacteria, erysipelotrichales, neisseriales, cw040, Chlorophyta, clostridiales, burkholderiales, Rickettsiales, bacteroidales, mycoplastiales, coriobacteriales Anaeroplasmatales, and Pseudanabaenales. The gut microbiota with differences at the family level include [paraprevotellaceae], corynebactriaceae, Veillonella CEAE, [odoribacterae], prevotellaceae, deferribacterae, staphylococcaceae, Rhodospirillaceae, anaeroplasmataceae, caulobacteraceae, streptococcaceae, dehalobactriaceae, christensenellaceae, desulfovibrionaceae, ruminococcaceae, F16 Bifidobacteriaceae, Helicobacteraceae, S24-7, and Pianococcacese; gut microbiota groups that differ at the genus level include [Prevotella], blautia, bilophila, Corynebacterium, Prevotella, Helicobacter, Lactococcus, rikenella, parabacteroides, anaeroplasma, Megasphaera, dehalobacterium, oscillospira, Clostridium, Streptococcus, Shigella, AF12, Desulfovibrio, and Candidatus_Arthromitus; the gut microbiota that produce differences at the species level Parabacteroides_distasonis, Mucispirillum_schaedleri, Alistipes_indistinctus, Bacteroides_uniformis, Corynebacterium_stationis, Lactobacillus_helveticus, Desulfovibrio_C21_c20, [Ruminococcus]_gnavus, Alistipes_finegoldii, Alistipes_onderdonkii, Sulfuricurvum_kujiense, Cellulomonas_uda, Butyricicoccus_pullicaecorum, Lactobacillus_vaginalis, Silene_vulgaris, Staphylococcus_sciuri, Helicobacter_hepaticus, Cetobacterium_somerae, Alistipes_massiliensis, Clostridium_cocleatum; by observing the gut microbiota with different levels of phyla and genus, it is found that there are 6 species of gut microbiota with callback effect at phyla level, namely, TM7, tenericutes, Chloroflex, cyanobacteria, acidobacteria, and WS6. There are 5 gut microbiota species with callback effect at the genus level, namely, [Prevotella], Helicobacter, Prevotella, Lactococcus, and anaeroplasma, as shown in Figure 5.

#### 3.3.6. Prediction of Metabolic Pathways in Microbiota Sample Communities

In order to identify the signaling pathway of Huangqin decoction in the treatment of DE, this study used picurst2 to perform functional analysis on the treatment group and identified 170 signaling pathways through enrichment, as shown in Table 3 below.

### 3.4. Network Pharmacology Analysis

After entering the keyword, “Scutellaria baicalensis, Paeonia alba, jujube and licorice” in the TCMSP database, 34 effective components of Scutellaria baicalensis, 8 effective components of Paeonia alba, 20 effective components of jujube, and 90 effective components of licorice were screened according to the screening conditions of OB ≥ 30% and DL ≥ 0.18. After merging and deleting multiple items, 141 components were obtained, as shown in Table 4. Using PubChem database (https://pubchem.ncbi.nlm.nih.gov/), obtain the SMILE standard structural formula of active ingredients and import it into the swisstargetprediction database (http://swisstargetprediction.ch/). Target prediction was carried out, duplicate targets were deleted, and a total of 265 targets related to active components were obtained.

To identify the main genes of Huangqin decoction's anti-DE (Table 5), Cytoscape 3.8.2 was used for visual analysis, and a protein-protein interaction network was constructed (Figure 6(c)). At the same time, the cytohubba plug-in was used to screen out the core targets. Combined with the score of the calculation method, the top 10 genes were considered as core genes (IL-6, TNF, TP53, IL1B, CASP3, JUN, PPARG, MAPK3, EGFR, and PTGS2) Table 6. GO annotation and KEGG pathway enrichment of the obtained potential target genes of Huangqin decoction against DE were performed by R language (Figures 6(d) and 6(e)). GO enrichment analysis showed that there was mainly positive regulation of nitric oxide biosynthetic process, response to ethanol, response to hypoxia, etc. According to KEGG enrichment analysis, the significantly affected pathways are bladder cancer, colorectal cancer, pancreatic cancer, leishmaniasis, hepatitis B, etc.

### 3.5. Integrating 16S rRNA Gene Sequencing and Network Pharmacology Analysis

In order to identify the signaling pathway of Huangqin decoction in the treatment of DE, this study used picurst2 to analyze the function of the treatment group and identified 170 signaling pathways through enrichment. Similar signaling pathways are followed by apoptosis (apoptosis), calcium signaling pathway (calcium signaling pathway), cell cycle-Caulobacter (cell cycle-Caulobacter), insulin signaling pathway (insulin signaling pathway), neurotrophin signaling pathway (neurotrophin signaling pathway), NOD-like receptor signaling pathway, and RIG-I-like receptor signaling pathway. Based on the core genes obtained from these seven signaling pathways and network pharmacology, an integrated network map of Huangqin decoction for the treatment of DE was drawn. As shown in Figure 7, the NOD-like receptor signaling pathway has the most significant node, and it has the strongest correlation with TNF and quercetin. Therefore, it is speculated that the mechanism of Huangqin decoction in the treatment of DE may be that the core component of Huangqin decoction, quercetin inhibits the expression of the TNF gene, thereby inhibiting the expression of NOD-like receptor signaling pathway and thereby achieving the therapeutic effect of the disease.

## 4. Discussion

This study combined network pharmacology and 16S rRNA sequencing. This study screened 156 active ingredients of Huangqin decoction in treating DE. Among them, quercetin as the core active ingredient, also known as quercetin, is a flavonoid compound with various biological activities. Quercetin and its derivatives are widely distributed in the plant kingdom, mostly in flowers, leaves, and fruits. Exist in the form of glycosides. It has expectorant, antitussive, antiasthmatic, anti-inflammatory, antiallergic, antispasmodic, cardiotonic, blood pressure lowering, coronary artery dilation, blood lipid lowering, antiarrhythmic, antiplatelet aggregation, antioxidant, antitumor, antioxidant, antidiabetic complications, and other pharmacological effects [18]. Ling and others showed that the mechanism of quercetin treatment in type 2 diabetic rats was that the substance activated the FGF21/MAPK signaling pathway in the pancreatic tissue increased the expression level of FGF21 and MAPK.

In contrast, the high level of FGF21 could significantly reduce the bodyweight of type 2 diabetic rats and accelerate the reabsorption of blood glucose, thereby lowering the level of blood sugar. *β* function of cells was maintained and played a role in improving insulin resistance. MAPK is the key kinase downstream of FGF21. This enzyme accelerates the absorption and utilization of sugars by increasing the expression of GLUT4, and the increase of insulin receptor sensitivity and insulin resistance is achieved through MAPK phosphorylation to achieve the effect of treating type 2 diabetes [19]. Mao Xiaoming et al. found that quercetin can inhibit the activity of aldose reductase in the diabetic kidney by measuring the urinary protein in the kidney tissue of experimental diabetic rats, and early application can prevent or delay the occurrence of diabetes [20]; in the research on the protective mechanism of quercetin on the kidneys of diabetic rats, it was found that quercetin can improve oxidative stress and have anti-inflammatory effects, thereby exerting a protective effect on early diabetes [21].

Tumor necrosis factor (TNF) has typical cytokine properties and is a major inflammatory factor and pleiotropic cellular regulatory protein. The excessive local release can trigger an inflammatory response and the body's immune response process. This factor is closely related to insulin and promotes insulin resistance by interfering with the insulin signal transduction pathway, resulting in the clinical manifestations of insulin resistance [22]. The KEGG signaling pathway enrichment results showed that the most prominent signaling pathway was NOD-like receptor signaling pathway. Relevant studies have shown that the innate immune system can recognize a variety of pathogenic microorganisms and is the body's first line of defense against pathogenic microorganisms. It recognizes invading pathogens by sensing pathogen-associated molecular patterns through specialized pattern recognition receptors (PRRs). They can be recognized by PRR-containing immune cells to initiate an immune response [23]. Among them, the NOD-like receptor family (NLR) in the cytoplasm, as one of the pattern recognition receptors, greatly influences the disease. NOD1 and NOD2 are members of the NODs subtypes of the NLRs family. NOD1 and NOD2 are cytoplasmic receptors for innate immunity that sense peptidoglycan from Gram-negative bacteria. Their functions have been extensively studied [24–26], revealing that they play a key role in host defense against pathogens such as Listeria monocytogenes, Helicobacter pylori, and Staphylococcus. In humans, dysregulation of NOD signaling pathways caused by mutations in NOD receptors, especially NOD2 receptors, is associated with inflammatory bowel disease. At the same time, related studies have found that NOD2 can recognize bacterial-derived cell muramyl dipeptide, which can induce the release of antimicrobial peptides and inflammatory signals required to maintain the homeostasis of intestinal flora, thereby protecting the host from bacterial invasion and thereby playing a role in preventing and treating diabetes. The expression of NOD2 is induced by bacterial components (lipopolysaccharide LPS), short-chain fatty acids (butyric acid), hormone vitamin D (1,25-dihydroxyvitamin D3), and proinflammatory cytokines (TNF-*α*), among others [27]. This is also consistent with the results of this experiment.

Some human diseases, including inflammatory bowel disease (IBD), diabetes, obesity, metabolic syndrome, fatty liver, and some neurological diseases, have been confirmed to be related to intestinal flora imbalance. The continuous exposure of intestinal tissue to microorganisms puts the intestinal mucosa in a state of physiological inflammation, where proinflammatory and anti-inflammatory responses are in balance to maintain body homeostasis [28]. If this relationship is unbalanced, it will lead to dysbiosis, where pathogenic bacteria dominate the commensal bacteria, causing damage to the intestinal epithelial barrier, bacterial invasion, and inflammation [29, 30]. To date, multiple studies have highlighted the important role of Nod2 in maintaining the balance between the microbial community and the host immune response [31, 32]. At the same time, the 16S rRNA results were consistent with it. In this study, we found 6 species of bacteria with callback effect at the phylum level, namely, TM7, Tenericutes, Chloroflexi, Cyanobacteria, Acidobacteria, and WS6. Among them, TM7 and Tenericutes are in the callback function. The most important value ranks among the phyla, and the research species related to diabetes are considered to be related to the inflammatory response. Tenericutes is the third dominant bacterial phylum in this study, which has been reported to be involved in the occurrence and development of diabetes. This study is closely related to the inflammatory response caused by high glucose, and the inhibition of Softwallia helps control the inflammatory response related to diabetes [33]. The proportions of TM7 were 2.48%, 5.55%, and 0.88%, respectively, and there was an obvious correction. TM7 was the sixth bacterial phylum in this study, which was confirmed to be positively correlated with the occurrence of inflammation in diabetes [34]; the genus level had a callback. There are 5 species of bacteria that act, namely, [Prevotella], Helicobacter, Prevotella, Lactococcus, and Anaeroplasma. Prevotella is the genus with the highest significant value in this study, and its level reduction is considered to be related to the inhibition of diabetes. These changes are related to the inflammatory responses [35, 36]. These changes indicate that Huangqin decoction can regulate the intestinal flora of diabetic mice. By regulating the abundance of bacteria, it protects the intestinal mucosa, improves the intestinal barrier function, and inhibits the inflammatory response generated in the high glucose state.

## 5. Conclusion

Through network pharmacology and 16S rRNA sequencing analysis, it was found that the mechanism of Huangqin decoction in the treatment of DE may be the prevention and treatment of the disease by inhibiting the expression of inflammatory factors in intestinal epithelial cells, thereby regulating the intestinal flora, but the exact molecular mechanism remains to need further verified.

## Figures and Tables

**Figure 1:** Influence of intestinal mucosal barrier integrity in DE model mice. Note: histomorphological changes in the cecum of db mice (H&E staining) (×20). (a) Intestinal mucosal structure of blank group; (b) intestinal mucosal structure of model group; (c) intestinal mucosal structure of Huangqin decoction group.

**Figure 2:** Immunohistochemistry of CD45 in the intestinal mucosa of DE mice. Note: immunohistochemical staining of cecal tissue of db mice to observe the changes of CD45 (×40); (a) CD45+ in the intestinal mucosa of the blank group; (b) CD45+ of intestinal mucosa in the model group; (c) effect of Huangqin decoction group on intestinal mucosa CD45+.

**Figure 3:** (a) Venn diagram of OTUs of gut microbiota in each group (K is blank group; M is model group; Q is Huangqin decoction group); (b–d) sparse curve of the intestinal flora of rat samples in each group (b), species accumulation curve (c), and rank-abundance curve (d).

**Figure 4:** Abundance distribution of intestinal flora in each group of rat samples at phylum (a) and genus (b) levels; analysis of the distribution of bacterial community structure in each group of rat samples (c).

**Figure 5:** Random forest plot of differential gut microbiota of samples in each group. Note: (a) phylum-level differential gut microbiota; (b) class-level differential gut microbiota; (c) order-level differential gut microbiota; (d) family-level differential gut microbiota; (e) genus-level differential gut microbiota; (f) species-level differential gut microbiota.

**Figure 6:** Network pharmacology analysis of Huangqin decoction in the treatment of DE. (a) Venn diagram of the intersection targets of Huangqin decoction and DE; (b) the component-target-disease interaction network of Huangqin decoction in the treatment of DE; (c) PPI network diagram of Huangqin decoction for anti-DE; (d, e) GO enrichment analysis and KEGG pathway enrichment analysis; *P* < 0.05 for all pathways.

**Figure 7:** Comprehensive network diagram of Huangqin decoction in the treatment of DE.

**Table 1:** Microbial diversity index of gut microbiota in each group.

Group	Chao1	Faith_pd	Goods_coverage	Observed_species	Pielou_e	Shannon	Simpson
Control group	2012.334	94.2689	0.9889872	1731.78	0.7317398	7.82702	0.9813612
Model group	1875.298	88.86688	0.9886164	1586.6	0.7124886	7.56511	0.9707218
Huangqin decoction group	1921.75	91.23156	0.989444	1669.04	0.7156288	7.692342	0.97627

**Table 2:** Statistical chart of difference analysis between groups.

Group 1	Group 2	Sample size	Permutations	Pseudo*F*	*P* value	*q* value
All	—	15	999	2.935413	0.001	—
K	M	10	999	2.408184	0.011	0.012
K	Q	10	999	3.450399	0.011	0.012
M	Q	10	999	2.986695	0.012	0.012

**Table 3:** Signal pathway of DE.

Pathway	Description
ko00010	Glycolysis/gluconeogenesis
ko00020	Citrate cycle (TCA cycle)
ko00030	Pentose phosphate pathway
ko00040	Pentose and glucuronate interconversions
ko00051	Fructose and mannose metabolism
ko00052	Galactose metabolism
ko00053	Ascorbate and aldarate metabolism
ko00061	Fatty acid biosynthesis
ko00071	Fatty acid metabolism
ko00072	Synthesis and degradation of ketone bodies
ko00100	Steroid biosynthesis
ko00120	Primary bile acid biosynthesis
ko00121	Secondary bile acid biosynthesis
ko00130	Ubiquinone and other terpenoid-quinone biosynthesis
ko00140	Steroid hormone biosynthesis
ko00190	Oxidative phosphorylation
ko00195	Photosynthesis
ko00196	Photosynthesis-antenna proteins
ko00230	Purine metabolism
ko00240	Pyrimidine metabolism
ko00250	Alanine, aspartate, and glutamate metabolism
ko00253	Tetracycline biosynthesis
ko00260	Glycine, serine, and threonine metabolism
ko00270	Cysteine and methionine metabolism
ko00280	Valine, leucine, and isoleucine degradation
ko00281	Geraniol degradation
ko00290	Valine, leucine, and isoleucine biosynthesis
ko00300	Lysine biosynthesis
ko00310	Lysine degradation
ko00311	Penicillin and cephalosporin biosynthesis
ko00312	Beta-lactam resistance
ko00330	Arginine and proline metabolism
ko00340	Histidine metabolism
ko00350	Tyrosine metabolism
ko00360	Phenylalanine metabolism
ko00361	Chlorocyclohexane and chlorobenzene degradation
ko00362	Benzoate degradation
ko00363	Bisphenol degradation
ko00364	Fluorobenzoate degradation
ko00380	Tryptophan metabolism
ko00400	Phenylalanine, tyrosine, and tryptophan biosynthesis
ko00410	Beta-alanine metabolism
ko00430	Taurine and hypotaurine metabolism
ko00440	Phosphonate and phosphinate metabolism
ko00450	Selenocompound metabolism
ko00460	Cyanoamino acid metabolism
ko00471	D-glutamine and D-glutamate metabolism
ko00472	D-arginine and D-ornithine metabolism
ko00473	D-alanine metabolism
ko00480	Glutathione metabolism
ko00500	Starch and sucrose metabolism
ko00510	N-glycan biosynthesis
ko00511	Other glycan degradation
ko00520	Amino sugar and nucleotide sugar metabolism
ko00521	Streptomycin biosynthesis
ko00523	Polyketide sugar unit biosynthesis
ko00524	Butirosin and neomycin biosynthesis
ko00531	Glycosaminoglycan degradation
ko00540	Lipopolysaccharide biosynthesis
ko00550	Peptidoglycan biosynthesis
ko00561	Glycerolipid metabolism
ko00562	Inositol phosphate metabolism
ko00564	Glycerophospholipid metabolism
ko00590	Arachidonic acid metabolism
ko00591	Linoleic acid metabolism
ko00600	Sphingolipid metabolism
ko00601	Glycosphingolipid biosynthesis-lacto and neolacto series
ko00620	Pyruvate metabolism
ko00621	Dioxin degradation
ko00622	Xylene degradation
ko00623	Toluene degradation
ko00624	Polycyclic aromatic hydrocarbon degradation
ko00625	Chloroalkane and chloroalkene degradation
ko00627	Aminobenzoate degradation
ko00630	Glyoxylate and dicarboxylate metabolism
ko00633	Nitrotoluene degradation
ko00640	Propanoate metabolism
ko00642	Ethylbenzene degradation
ko00643	Styrene degradation
ko00650	Butanoate metabolism
ko00660	C5-branched dibasic acid metabolism
ko00670	One carbon pool by folate
ko00680	Methane metabolism
ko00710	Carbon fixation in photosynthetic organisms
ko00720	Carbon fixation pathways in prokaryotes
ko00730	Thiamine metabolism
ko00740	Riboflavin metabolism
ko00750	Vitamin B6 metabolism
ko00760	Nicotinate and nicotinamide metabolism
ko00770	Pantothenate and CoA biosynthesis
ko00780	Biotin metabolism
ko00785	Lipoic acid metabolism
ko00790	Folate biosynthesis
ko00791	Atrazine degradation
ko00830	Retinol metabolism
ko00860	Porphyrin and chlorophyll metabolism
ko00900	Terpenoid backbone biosynthesis
ko00903	Limonene and pinene degradation
ko00906	Carotenoid biosynthesis
ko00908	Zeatin biosynthesis
ko00909	Sesquiterpenoid biosynthesis
ko00910	Nitrogen metabolism
ko00920	Sulfur metabolism
ko00930	Caprolactam degradation
ko00941	Flavonoid biosynthesis
ko00943	Isoflavonoid biosynthesis
ko00960	Tropane, piperidine, and pyridine alkaloid biosynthesis
ko00965	Betalain biosynthesis
ko00970	Aminoacyl-tRNA biosynthesis
ko00980	Metabolism of xenobiotics by cytochrome P450
ko00983	Drug metabolism-other enzymes
ko01040	Biosynthesis of unsaturated fatty acids
ko01051	Biosynthesis of ansamycins
ko01053	Biosynthesis of siderophore group nonribosomal peptides
ko01055	Biosynthesis of vancomycin group antibiotics
ko01056	Biosynthesis of type II polyketide backbone
ko02010	ABC transporters
ko02020	Two-component system
ko02030	Bacterial chemotaxis
ko02040	Flagellar assembly
ko02060	Phosphotransferase system (PTS)
ko03008	Ribosome biogenesis in eukaryotes
ko03010	Ribosome
ko03013	RNA transport
ko03015	mRNA surveillance pathway
ko03018	RNA degradation
ko03020	RNA polymerase
ko03030	DNA replication
ko03040	Spliceosome
ko03050	Proteasome
ko03060	Protein export
ko03070	Bacterial secretion system
ko03410	Base excision repair
ko03420	Nucleotide excision repair
ko03430	Mismatch repair
ko03440	Homologous recombination
ko03450	Nonhomologous end-joining
ko04020	Calcium signaling pathway
ko04112	Cell cycle-Caulobacter
ko04113	Meiosis-yeast
ko04122	Sulfur relay system
ko04141	Protein processing in endoplasmic reticulum
ko04142	Lysosome
ko04144	Endocytosis
ko04145	Phagosome
ko04146	Peroxisome
ko04210	Apoptosis
ko04310	Wnt signaling pathway
ko04621	NOD-like receptor signaling pathway
ko04622	RIG-I-like receptor signaling pathway
ko04626	Plant-pathogen interaction
ko04722	Neurotrophin signaling pathway
ko04910	Insulin signaling pathway
ko04962	Vasopressin-regulated water reabsorption
ko04974	Protein digestion and absorption
ko05010	Alzheimer's disease
ko05012	Parkinson's disease
ko05100	Bacterial invasion of epithelial cells
ko05110	Vibrio cholerae infection
ko05111	Vibrio cholerae pathogenic cycle
ko05120	Epithelial cell signaling in Helicobacter pylori infection
ko05130	Pathogenic Escherichia coli infection
ko05131	Shigellosis
ko05143	African trypanosomiasis
ko05145	Toxoplasmosis
ko05146	Amoebiasis
ko05150	Staphylococcus aureus infection
ko05200	Pathways in cancer
ko05322	Systemic lupus erythematosus
ko05410	Hypertrophic cardiomyopathy (HCM)

**Table 4:** Effective ingredients of HQD.

MOL ID	Ingredient	OB (%)	DL	Source
MOL000422	Kaempferol	41.88224954	0.24066	Licorice, white peony root
MOL000359	Sitosterol	36.91390583	0.7512	Licorice, Scutellaria baicalensis, white peony root
MOL000098	Quercetin	46.43334812	0.27525	Jujube, licorice
MOL000211	Mairin	55.37707338	0.7761	Jujube, licorice, white peony root
MOL000358	Beta-sitosterol	36.91390583	0.75123	Jujube, Scutellaria baicalensis, white peony root
MOL000449	Stigmasterol	43.82985158	0.75665	Jujube, Scutellaria baicalensis
MOL000492	(+)-catechin	54.82643405	0.24164	Jujube, white peony root
MOL000096	(-)-catechin	49.6763868	0.24162	Jujube
MOL000627	Stepholidine	33.10625074	0.54083	
MOL000787	Fumarine	59.26250458	0.82694	
MOL001454	Berberine	36.86124504	0.77665	
MOL001522	S-coclaurine	42.35064217	0.23518	
MOL002773	Beta-carotene	37.18433337	0.58358	
MOL004350	Ruvoside_qt	36.12101953	0.75671	
MOL007213	Nuciferin	34.43102883	0.40475	
MOL012921	Stepharine	31.54786691	0.33376	
MOL012946	Zizyphus saponin I_qt	32.69113507	0.61923	
MOL012976	Coumestrol	32.48702929	0.33733	
MOL012981	Daechuine S7	44.81774487	0.82806	
MOL012986	Jujubasaponin V_qt	36.98963109	0.63448	
MOL012992	Mauritine D	89.12509381	0.45286	
MOL000263	Oleanolic acid	29.02	0.76	
MOL000354	Isorhamnetin	49.60437705	0.306	Licorice
MOL003656	Lupiwighteone	51.63569181	0.36739	
MOL004808	Glyasperin B	65.22438608	0.43851	
MOL004810	Glyasperin F	75.83680013	0.53514	
MOL004811	Glyasperin C	45.56380662	0.39947	
MOL004820	Kanzonols W	50.48007599	0.51704	
MOL004824	(2S)-6-(2,4-dihydroxyphenyl)-2-(2-hydroxypropan-2-yl)-4-methoxy-2,3-dihydrofuro[3,2-g]chromen-7-one	60.25040908	0.63433	
MOL004827	Semilicoisoflavone B	48.77755194	0.54732	
MOL004828	Glepidotin A	44.72187465	0.34685	
MOL004829	Glepidotin B	64.46292386	0.34485	
MOL004849	3-(2,4-Dihydroxyphenyl)-8-(1,1-dimethylprop-2-enyl)-7-hydroxy-5-methoxy-coumarin	59.62247498	0.42894	
MOL004855	Licoricone	63.57845938	0.4712	
MOL004856	Gancaonin A	51.07519107	0.40378	
MOL004857	Gancaonin B	48.79440201	0.44924	
MOL004864	5,7-Dihydroxy-3-(4-methoxyphenyl)-8-(3-methylbut-2-enyl)chromone	30.48877673	0.41002	
MOL004879	Glycyrin	52.60657166	0.47466	
MOL004883	Licoisoflavone	41.61021885	0.41646	
MOL004884	Licoisoflavone B	38.92870888	0.54714	
MOL004885	Licoisoflavanone	52.46624706	0.54488	
MOL004904	Licopyranocoumarin	80.36001331	0.6535	
MOL004959	1-Methoxyphaseollidin	36.56537233	0.32291	
MOL004966	3′-Hydroxy-4′-O-methylglabridin	43.71495141	0.57406	
MOL004974	3′-Methoxyglabridin	46.16150929	0.57393	
MOL005000	Gancaonin G	60.43520506	0.39404	
MOL005001	Gancaonin H	50.10372327	0.78416	
MOL005007	Glyasperins M	72.67080984	0.59274	
MOL005008	Glycyrrhiza flavonol A	41.27527733	0.59512	
MOL000497	Licochalcone a	40.78965199	0.28517	
MOL004328	Naringenin	59.29389773	0.21128	
MOL004903	Liquiritin	65.69011165	0.73893	
MOL000392	Formononetin	69.67388061	0.21202	
MOL000500	Vestitol	74.65518912	0.20935	
MOL001792	DFV	32.76272375	0.18316	
MOL002565	Medicarpin	49.21981761	0.3351	
MOL003896	7-Methoxy-2-methyl isoflavone	42.56474148	0.19946	
MOL004835	Glypallichalcone	61.59706227	0.18993	
MOL004941	(2R)-7-hydroxy-2-(4-hydroxyphenyl)chroman-4-one	71.12298901	0.18303	
MOL004957	HMO	38.3654238	0.21067	
MOL004978	2-[(3R)-8,8-dimethyl-3,4-dihydro-2H-pyrano[6,5-f]chromen-3-yl]-5-methoxyphenol	36.21429208	0.52122	
MOL000239	Jaranol	50.82881677	0.29148	
MOL001484	Inermine	75.18306038	0.53754	
MOL004806	Euchrenone	30.28726099	0.57386	
MOL004815	(E)-1-(2,4-dihydroxyphenyl)-3-(2,2-dimethylchromen-6-yl)prop-2-en-1-one	39.61685537	0.35077	
MOL004833	Phaseolinisoflavan	32.00810772	0.44538	
MOL004866	2-(3,4-Dihydroxyphenyl)-5,7-dihydroxy-6-(3-methylbut-2-enyl)chromone	44.15196126	0.41482	
MOL004891	Shinpterocarpin	80.29527688	0.72746	
MOL004908	Glabridin	53.24514328	0.46967	
MOL004910	Glabranin	52.89565508	0.31208	
MOL004911	Glabrene	46.26685721	0.43902	
MOL004912	Glabrone	52.51217419	0.49645	
MOL004915	Eurycarpin A	43.27728425	0.37429	
MOL004945	(2S)-7-hydroxy-2-(4-hydroxyphenyl)-8-(3-methylbut-2-enyl)chroman-4-one	36.56537233	0.32291	
MOL004961	Quercetin der.	46.4493884	0.3343	
MOL004980	Inflacoumarin A	39.70909598	0.32613	
MOL004989	6-Prenylated eriodictyol	39.22383018	0.41259	
MOL004991	7-Acetoxy-2-methylisoflavone	38.92333105	0.26217	
MOL004993	8-Prenylated eriodictyol	53.79476318	0.40383	
MOL005003	Licoagrocarpin	58.81390287	0.58498	
MOL005012	Licoagroisoflavone	57.28224098	0.48679	
MOL005016	Odoratin	49.94821817	0.30487	
MOL005020	Dehydroglyasperins C	53.82326014	0.37006	
MOL000417	Calycosin	47.75182783	0.24278	
MOL004838	8-(6-Hydroxy-2-benzofuranyl)-2,2-dimethyl-5-chromenol	58.43728091	0.38106	
MOL004863	3-(3,4-Dihydroxyphenyl)-5,7-dihydroxy-8-(3-methylbut-2-enyl)chromone	66.37125046	0.41392	
MOL002311	Glycyrol	90.77578223	0.66819	
MOL004805	(2S)-2-[4-hydroxy-3-(3-methylbut-2-enyl)phenyl]-8,8-dimethyl-2,3-dihydropyrano[2,3-f]chromen-4-one	31.78703353	0.72403	
MOL004814	Isotrifoliol	31.94478724	0.42422	
MOL004841	Licochalcone B	76.75735485	0.1935	
MOL004848	Licochalcone G	49.25496332	0.32325	
MOL004898	(E)-3-[3,4-dihydroxy-5-(3-methylbut-2-enyl)phenyl]-1-(2,4-dihydroxyphenyl)prop-2-en-1-one	46.26792256	0.3062	
MOL004907	Glyzaglabrin	61.06888631	0.35347	
MOL004924	(-)-Medicocarpin	40.99397199	0.95059	
MOL004935	Sigmoidin-B	34.88108616	0.41455	
MOL004948	Isoglycyrol	44.69922568	0.83845	
MOL004949	Isolicoflavonol	45.16999058	0.41859	
MOL004988	Kanzonol F	32.46833364	0.89364	
MOL004990	7,2′,4′-trihydroxy-5-methoxy-3-arylcoumarin	83.71436744	0.27136	
MOL005017	Phaseol	78.76621925	0.57867	
MOL005018	Xambioona	54.84916242	0.87419	
MOL004913	1,3-Dihydroxy-9-methoxy-6-benzofurano[3,2-c]chromenone	48.14154235	0.42831	
MOL004914	1,3-Dihydroxy-8,9-dimethoxy-6-benzofurano[3,2-c]chromenone	62.90135486	0.52759	
MOL004985	Icos-5-enoic acid	30.70294255	0.19725	
MOL004996	Gadelaidic acid	30.70294255	0.19725	
MOL004882	Licocoumarone	33.21085068	0.3568	
MOL001789	Isoliquiritigenin	85.32	0.15	
MOL004804	18Beta-glycyrrhetinic acid	22.05	0.74	
MOL000073	Ent-epicatechin	48.95984114	0.24162	Scutellaria baicalensis
MOL000173	Wogonin	30.68456706	0.22942	
MOL000228	(2R)-7-hydroxy-5-methoxy-2-phenylchroman-4-one	55.23317389	0.20163	
MOL000525	Norwogonin	39.40397184	0.20723	
MOL000552	5,2′-Dihydroxy-6,7,8-trimethoxyflavone	31.71246493	0.35462	
MOL001458	Coptisine	30.671852	0.85647	
MOL001490	Bis[(2S)-2-ethylhexyl] benzene-1,2-dicarboxylate	43.59332547	0.34531	
MOL001689	Acacetin	34.97357273	0.24082	
MOL002714	Baicalein	33.51891869	0.20888	
MOL002879	Diop	43.59332547	0.39247	
MOL002897	Epiberberine	43.09233228	0.7761	
MOL002909	5,7,2,5-Tetrahydroxy-8,6-dimethoxyflavone	33.81582599	0.44739	
MOL002910	Carthamidin	41.15096273	0.24189	
MOL002913	Dihydrobaicalin_qt	40.03778103	0.20722	
MOL002914	Eriodyctiol (flavanone)	41.35042713	0.2436	
MOL002915	Salvigenin	49.06592606	0.33279	
MOL002917	5,2′,6′-Trihydroxy-7,8-dimethoxyflavone	45.04742802	0.33057	
MOL002925	5,7,2′,6′-Tetrahydroxyflavone	37.01348688	0.24382	
MOL002927	Skullcapflavone II	69.51043398	0.4379	
MOL002928	Oroxylin a	41.367569	0.23233	
MOL002932	Panicolin	76.25704989	0.2915	
MOL002933	5,7,4′-Trihydroxy-8-methoxyflavone	36.56200469	0.26666	
MOL002934	Neobaicalein	104.3446052	0.43917	
MOL002937	Dihydrooroxylin	66.06173872	0.23057	
MOL008206	Moslosooflavone	44.08795959	0.25331	
MOL010415	11,13-Eicosadienoic acid, methyl ester	39.27534422	0.2289	
MOL012245	5,7,4′-trihydroxy-6-methoxyflavanone	36.62688628	0.26833	
MOL012246	5,7,4′-Trihydroxy-8-methoxyflavanone	74.23522001	0.26479	
MOL012266	Rivularin	37.94023355	0.3663	
MOL002776	Baicalin	40.12	0.75	
MOL001918	Paeoniflorgenone	87.59312084	0.36678	White peony root
MOL001919	(3S,5R,8R,9R,10S,14S)-3,17-dihydroxy-4,4,8,10,14-pentamethyl-2,3,5,6,7,9-hexahydro-1H-cyclopenta[a]phenanthrene-15,16-dione	43.55620167	0.53276	
MOL001924	Paeoniflorin	53.87037516	0.78709	

**Table 5:** Target information of DE in network pharmacology.

No.	Gene names	Protein names	Uniprot ID
1	TGFB1	Transforming growth factor beta-1 proprotein [cleaved into: latency-associated peptide	P01137
2	SLC6A4	Sodium-dependent serotonin transporter	P31645
3	PTGS2	Prostaglandin G/H synthase 2	P35354
4	PTGS1	Prostaglandin G/H synthase 1	P23219
5	PRKCA	Protein kinase C alpha type	P17252
6	PRKACA	cAMP-dependent protein kinase catalytic subunit alpha	P17612
7	PON1	Serum paraoxonase/arylesterase 1	P27169
8	PIK3CG	Phosphatidylinositol 4,5-bisphosphate 3-kinase catalytic subunit gamma isoform	P48736
9	OPRM1	Mu-type opioid receptor	P35372
10	JUN	Transcription factor AP-1	P05412
11	HTR2A	5-Hydroxytryptamine receptor 2A	P28223
12	HSP90AA1	Heat shock protein HSP 90-alpha	P07900
13	CASP9	Caspase-9	P55211
14	CASP8	Caspase-8	Q14790
15	CASP3	Caspase-3	P42574
16	BCL2	Apoptosis regulator Bcl-2	P10415
17	BAX	Apoptosis regulator BAX	Q07812
18	ADRB2	Beta-2 adrenergic receptor	P07550
19	NR3C2	Mineralocorticoid receptor	P08235
20	XDH	Xanthine dehydrogenase/oxidase [includes: xanthine dehydrogenase	P47989
21	VCAM1	Vascular cell adhesion protein 1	P19320
22	TNF	Tumor necrosis factor	P01375
23	STAT1	Signal transducer and activator of transcription 1-alpha/beta	P42224
24	SLPI	Antileukoproteinase	P03973
25	SLC2A4	Solute carrier family 2, facilitated glucose transporter member 4	P14672
26	SELE	E-selectin	P16581
27	RELA	Transcription factor p65	Q04206
28	PRSS1	Trypsin-1	P07477
29	PPARG	Peroxisome proliferator-activated receptor gamma	Q08209
30	NOS3	Nitric oxide synthase, endothelial	P37231
31	NOS2	Nitric oxide synthase, inducible	Q14994
32	MMP1	Interstitial collagenase	O75469
33	MAPK8	Mitogen-activated protein kinase 8	P29474
34	INSR	Insulin receptor	P35228
35	IKBKB	Inhibitor of nuclear factor kappa-B kinase subunit beta	P03956
36	ICAM1	Intercellular adhesion molecule 1	P45983
37	HMOX1	Heme oxygenase 1	P06213
38	GSTM1	Glutathione S-transferase Mu 1	O14920
39	F7	Coagulation factor VII	P05362
40	F2	Prothrombin	P09601
41	DPP4	Dipeptidyl peptidase 4	P09488
42	CYP3A4	Cytochrome P450 3A4	P08709
43	CYP1A1	Cytochrome P450 1A1	P00734
44	CDK1	Cyclin-dependent kinase 1	P27487
45	AR	Androgen receptor	P08684
46	ALOX5	Polyunsaturated fatty acid 5-lipoxygenase	P04798
47	AKT1	RAC-alpha serine/threonine-protein kinase	P06493
48	AHR	Aryl hydrocarbon receptor	P10275
49	ACHE	Acetylcholinesterase	P09917
50	ESR1	Estrogen receptor	P31749
51	IL6	Interleukin-6	P35869
52	CD14	Monocyte differentiation antigen CD14	P22303
53	FASN	Fatty acid synthase	P19793
54	TP53	Cellular tumor antigen p53	P03372
55	THBD	Thrombomodulin	P18428
56	SPP1	Osteopontin	P05231
57	SOD1	Superoxide dismutase [Cu-Zn]	P08571
58	SERPINE1	Plasminogen activator inhibitor 1	P49327
59	RUNX2	Runt-related transcription factor 2	P04637
60	RB1	Retinoblastoma-associated protein	P07204
61	RAF1	RAF protooncogene serine/threonine-protein kinase	P10451
62	PTEN	Phosphatidylinositol 3,4,5-trisphosphate 3-phosphatase and dual-specificity protein phosphatase PTEN	P00441
63	PRKCB	Protein kinase C beta type	P05121
64	PPARD	Peroxisome proliferator-activated receptor delta	Q13950
65	PPARA	Peroxisome proliferator-activated receptor alpha	P06400
66	PLAU	Urokinase-type plasminogen activator	P04049
67	PLAT	Tissue-type plasminogen activator	P60484
68	PARP1	Poly [ADP-ribose] polymerase 1	P05771
69	ODC1	Ornithine decarboxylase	Q03181
70	NQO1	NAD	Q07869
71	NFKBIA	NF-kappa-B inhibitor alpha	P00749
72	NFE2L2	Nuclear factor erythroid 2-related factor 2	P00750
73	NCF1	Neutrophil cytosol factor 1	P09874
74	MYC	Myc protooncogene protein	P11926
75	MPO	Myeloperoxidase	P15559
76	MMP9	Matrix metalloproteinase-9	P25963
77	MMP3	Stromelysin-1	Q16236
78	MMP2	72 kDa type IV collagenase	P01106
79	MGAM	Maltase-glucoamylase, intestinal [includes: maltase	P05164
80	MAPK1	Mitogen-activated protein kinase 1	P14780
81	IL2	Interleukin-2	P08254
82	IL1B	Interleukin-1 beta	P08253
83	IL1A	Interleukin-1 alpha	O43451
84	IL10	Interleukin-10	P28482
85	IGFBP3	Insulin-like growth factor-binding protein 3	P60568
86	IGF2	Insulin-like growth factor II	P01584
87	IFNG	Interferon gamma	P01583
88	HSPB1	Heat shock protein beta-1	P22301
89	HSPA5	Endoplasmic reticulum chaperone BiP	P17936
90	HK2	Hexokinase-2	P01344
91	HIF1A	Hypoxia-inducible factor 1-alpha	P01579
92	GJA1	Gap junction alpha-1 protein	P04792
93	FOS	Protooncogene c-Fos	P11021
94	F3	Tissue factor	P52789
95	ERBB3	Receptor tyrosine-protein kinase erbB-3	Q16665
96	ERBB2	Receptor tyrosine-protein kinase erbB-2	P17302
97	EGFR	Epidermal growth factor receptor	P01100
98	CXCL8	Interleukin-8	P13726
99	CXCL10	C-X-C motif chemokine 10	P00742
100	CTSD	Cathepsin D	P21860
101	CRP	C-reactive protein [cleaved into: C-reactive protein]	P04626
102	CLDN4	Claudin-4	P00533
103	CHEK2	Serine/threonine-protein kinase Chk2	Q01094
104	CDKN1A	Cyclin-dependent kinase inhibitor 1	P10145
105	CD40LG	CD40 ligand	P19875
106	CCND1	G1/S-specific cyclin-D1	P02778
107	CCL2	C-C motif chemokine 2	P07339
108	CAV1	Caveolin-1	P02741
109	BIRC5	Baculoviral IAP repeat-containing protein 5	P02461
110	AKR1B1	Aldo-keto reductase family 1 member B1	O96017
111	ACACA	Acetyl-CoA carboxylase 1	P38936
112	ADRB1	Beta-1 adrenergic receptor	P29965
113	ADRA2A	Alpha-2A adrenergic receptor	P24385
114	HTR2C	5-Hydroxytryptamine receptor 2C	P13500
115	DRD4	D	Q03135
116	ADRA2B	Alpha-2B adrenergic receptor	O15392
117	PDE4D	cAMP-specific 3′,5′-cyclic phosphodiesterase 4D	Q07817
118	KDR	Vascular endothelial growth factor receptor 2	P15121
119	HTR3A	5-Hydroxytryptamine receptor 3A	Q13085
120	CTNNB1	Catenin beta-1	P21397
121	DRD2	D	P08588
122	ESR2	Estrogen receptor beta	P35968
123	CDK2	Cyclin-dependent kinase 2	P35222
124	PTPN1	Tyrosine-protein phosphatase nonreceptor type 1	P55210
125	OLR1	Oxidized low-density lipoprotein receptor 1	P14416
126	MAPK14	Mitogen-activated protein kinase 14	P20813
127	GSK3B	Glycogen synthase kinase-3 beta	Q92731
128	SIRT1	NAD-dependent protein deacetylase sirtuin-1	P24941
129	MT-ND6	NADH-ubiquinone oxidoreductase chain 6	P18031
130	IL4	Interleukin-4	P78380
131	STAT3	Signal transducer and activator of transcription 3	Q16539
132	CDK4	Cyclin-dependent kinase 4	P49841
133	JAK2	Tyrosine-protein kinase JAK2	Q96EB6
134	SLC2A1	Solute carrier family 2, facilitated glucose transporter member 1	P03923
135	MAPK10	Mitogen-activated protein kinase 10	P05112
136	SREBF1	Sterol regulatory element-binding protein 1	P40763
137	SOAT1	Sterol O-acyltransferase 1	P11802
138	MTTP	Microsomal triglyceride transfer protein large subunit	O60674
139	MAPK3	Mitogen-activated protein kinase 3	P11166
140	LDLR	Low-density lipoprotein receptor	P53779
141	HMGCR	3-Hydroxy-3-methylglutaryl-coenzyme A reductase	P36956
142	GSR	Glutathione reductase, mitochondrial	P55157
143	CYP19A1	Aromatase	P27361
144	BAD	Bcl2-associated agonist of cell death	P01130
145	APOB	Apolipoprotein B-100	P04035
146	ADIPOQ	Adiponectin	P00390
147	CAT	Catalase	P11511
148	UGT1A1	UDP-glucuronosyltransferase 1A1	P23141
149	HSD11B2	Corticosteroid 11-beta-dehydrogenase isozyme 2	Q92934
150	CYP2E1	Cytochrome P450 2E1	P04114
151	KCNMA1	Calcium-activated potassium channel subunit alpha-1	Q15848
152	FN1	Fibronectin	P33527
153	PRKCD	Protein kinase C delta type	P04040
154	FASLG	Tumor necrosis factor ligand superfamily member 6	P22309
155	CYCS	Cytochrome c	P05181
156	CYP2C9	Cytochrome P450 2C9	P02751

**Table 6:** CytoHubba key genes screened.

Gene symbol	Rank methods in CytoHubba									
	MCC	MNC	Degree	EPC	BottleNeck	EcCentricity	Closeness	Radiality	Betweenness	Stress
IL-6	9.22*E*+13	123	246	25.989	24	0.5	139	3.82581	1344.73372	83272
TNF	9.22*E*+13	117	234	25.101	1	0.5	136	3.7871	874.01279	78512
TP53	9.22*E*+13	116	232	23.732	2	0.5	135.5	3.78065	771.82047	70320
IL1B	9.22*E*+13	110	220	25.059	1	0.33333	132.33333	3.73548	506.5106	50800
CASP3	9.22*E*+13	106	212	23.827	5	0.33333	130.33333	3.70968	520.91581	53936
JUN	9.22*E*+13	104	208	23.701	1	0.33333	129.33333	3.69677	383.48979	42960
PPARG	9.22*E*+13	101	202	23.55	1	0.33333	127.83333	3.67742	309.07813	36088
MAPK3	9.22*E*+13	99	198	24.044	37	0.5	127	3.67097	555.13067	49336
EGFR	9.22*E*+13	98	196	23.689	1	0.5	126.5	3.66452	354.85078	40368
PTGS2	9.22*E*+13	95	190	23.301	1	0.5	125	3.64516	700.314	59256

## Data Availability

The data used to support this study are available from the corresponding author upon request.

## Abbreviations

DE: Diabetic enteritis
GO: Gene Ontology
KEGG: Kyoto Encyclopedia of Genes and Genomes
TCMSP: Traditional Chinese medicine systems pharmacology.
